# The Identification of Key Genes and Biological Pathways in Heart Failure by Integrated Bioinformatics Analysis

**DOI:** 10.1155/2021/3859338

**Published:** 2021-11-26

**Authors:** Qianhong Yang, Xiaolu Bai, Xiang Li, Wei Hu

**Affiliations:** ^1^Department of Geriatrics, Minhang Hospital, Fudan University, 170 Xinsong Road, Shanghai 201199, China; ^2^Department of Cardiology, Minhang Hospital, Fudan University, 170 Xinsong Road, Shanghai 201199, China; ^3^Department of Critical Care Medicine, Minhang Hospital, Fudan University, 170 Xinsong Road, Shanghai 201199, China

## Abstract

**Purpose:**

Heart failure (HF) is a clinical syndrome caused by ventricular insufficiency. In order to further explore the biomarkers related to HF, we apply the high-throughput database.

**Materials and Methods:**

The GSE21610 was applied for the differentially expressed gene (DEG) analysis. The Database for Annotation, Visualization, and Integrated Discovery (DAVID) was performed to assess Gene ontology (GO) and the Kyoto Encyclopedia of Genes and Genomes (KEGG) analyses. The Gene Set Enrichment Analysis (GSEA) was used for gene expression profile GSE21610. The Protein-Protein Interaction (PPI) network and modules were also constructed for research. These hub gene function pathways were estimated in HF progression.

**Result:**

We have identified 434 DEGs in total, including 304 downregulated DEGs and 130 upregulated DEGs. GO and KEGG illustrated that DEGs in HF were significantly enriched in G protein-coupled receptor binding, peroxisome, and cAMP signaling pathway. GSEA results showed gene set GSE21610 was gathered in lipid digestion, defense response to fungus, and intestinal lipid absorption. Finally, through analyzing the PPI network, we screened hub genes CDH1, TFRC, CCL2, BUB1B, and CD19 by the Cytoscape software.

**Conclusion:**

This study uses a series of bioinformatics technologies to obtain hug genes and key pathways related to HF. These analysis results provide us with new ideas for finding biomarkers and treatment methods for HF.

## 1. Background

Heart failure (HF) is generally a syndrome in which the heart cannot pump out the same venous return and the blood supply needed for body tissue metabolism [1]. Data for 2020 showed that there were approximately 22.5 million HF patients worldwide, with a mortality rate as high as 50% [2]. Clinically, HF is divided into two types: acute and chronic. Chronic HF has a slow onset, usually manifested as an enlarged or thickened heart, and acute HF manifests as severe myocardial damage and arrhythmia [3]. Cardiomyopathy, heart overload, myocardial inflammation, and other cardiovascular diseases can induce the occurrence of HF, especially in patients with a history of coronary heart disease and hypertension [4]. Generally, different treatment methods are adopted according to the different severities of the patients, including not only drug treatments, such as RAAS inhibitors, *β*-receptor antagonists, and nitrate drugs, but also surgery and traditional Chinese medicine treatments [5]. However, because HF is a progressive disease, only 50% of patients have a good prognosis after targeted treatment, and many advanced patients still have a poor prognosis [6]. Therefore, the discovery of effective biomarkers for the treatment of HF is very important.

High-throughput gene microarray analysis is the latest technology, which can detect multiple chips at the same time and minimize system errors and has extremely high sensitivity [7]. At present, this technology has been widely used in the research of diseases, which has opened up a milestone in the field of genomics research on human diseases, making whole-genome resequencing possible [8–11]. In the process of this research on HF, based on this technology, we can detect and explore the gene expression of HF at the molecular level.

In this study, we downloaded GSE21610 based on the Gene Expression Omnibus (GEO) database and selected 68 samples as the basis for analysis. First, differentially expressed genes (DEGs) were analyzed from the samples by GEO2R, and then, the functional enrichment of DEGs in Gene Ontology (GO) and Kyoto Encyclopedia of Genes and Genomes (KEGG) was analyzed with the help of Database for Annotation, Visualization, and Integrated Discovery (DAVID). Subsequently, the entire sample was analyzed by Gene Set Enrichment Analysis (GSEA) for biological process (BP) enrichment. Next, Search Tool for the Retrieval of Interacting Genes (STRING) and Cytoscape were used to construct a Protein-Protein Interaction (PPI) network and screen out the hub genes. Finally, in order to clarify the roles of the hub genes in HF, the levels of the two groups of 68 samples were compared and analyzed. The above bioinformatics results will deepen our understanding of HF and find new treatment options.

## 2. Materials and Methods

### 2.1. Microarray Data Processing

The GEO database contains storage chips, next-generation sequencing, and other high-throughput sequencing data, which can be used to retrieve experimental sequencing data uploaded by others [12]. We downloaded GSE21610 data set from the GEO (https://www.ncbi.nlm.nih.gov/geo/) database. The data set contains a total of 68 sample data, from which 8 groups of disease-free control myocardium and 30 paired samples of VAD (ventricular assistance device) support myocardium with previous HF were collected as the sample data for this study.

### 2.2. Identification of DEGs

Based on the online analysis software of GEO2R (https://www.ncbi.nlm.nih.gov/geo/geo2r/) in the GEO database, we analyzed 8 groups of control samples and 30 paired samples of VAD samples. According to the standard, we used FC > 2 as the screening criterion for upregulation of DEGs and FC < 0.5 for downregulation of DEGs. When *P* < 0.01, it had statistical significance. The final selected DEGs were displayed through the volcano map.

### 2.3. Enrichment Analysis of GO Term and KEGG Pathways of DEGs

GO is a term used to describe the features of genes and gene products, including three parts: BP, cellular component (CC), and molecular function (MF) [13]. KEGG is a gene product analysis in cellular metabolic pathways and often used to analyze metabolic pathways [14]. In this study, to clarify the biological functions of DEGs, based on the DAVID (https://david.ncifcrf.gov/), we performed enrichment analysis of DEGs in GO and KEGG. The results obtained were displayed in histograms and scatter plots.

### 2.4. GSEA of 68 Samples

GSEA is a calculation method used to test whether a predefined gene set shows a significant consistent difference between two biological states [15]. In this study, we tested the enrichment of genes in 8 groups of controls and 30 paired samples of VAD cases in BP through GSEA and set *P* < 0.05 as the standard.

### 2.5. Construction of the PPI Network and Identification of Hub Genes

In order to find the hub genes in HF, we integrated the cross-correlation of DEGs through the STRING (https://string-db.org/) database. Later, with the help of the Cytoscape (http://www.cytoscape.org/) software, a PPI network of DEGs was constructed, which was helpful for systematic research on the molecular mechanisms of diseases and therapeutic targets [16]. Finally, for the sake of screening out the hub genes from the PPI network according to the degree value. Genes with a degree ≥ 12 were defined as hub genes.

## 3. Results

### 3.1. Screening of DEGs

The samples in this study included 8 groups of control and 30 paired samples of VAD cases. Based on the GEO2R analysis of these samples and the set screening conditions, we obtained a total of 434 DEGs, of which 304 were downregulated DEGs and 130 upregulated DEGs (Figure 1).

### 3.2. Enrichment Analysis of GO Term and KEGG Pathways of Upregulated DEGs

Figure 2(a) is the enrichment analysis result of upregulated DEGs in GO. It was seen that upregulated DEGs were in BP associated with the regulation of aldosterone biosynthetic, very long-chain fatty acid catabolic, sterol metabolic, and estrogen biosynthetic processes. In CC, the upregulated DEGs were related to Golgi lumen, intracellular organelle lumen, SCF ubiquitin ligase complex, mitochondrial outer membrane, etc. In MF, these DEGs were also related to cell adhesion mediator activity, histone demethylase activity, G protein-coupled receptor binding, peptidase inhibitor activity, and cell-cell adhesion mediator activity.  Figure 2(b) shows the top 5 KEGG pathways enriched by upregulated DEGs, namely, peroxisome, African trypanosomiasis, primary immunodeficiency, ABC transporters, and regulation of lipolysis in adipocytes.

### 3.3. Enrichment Analysis of GO Term and KEGG Pathways of Downregulated DEGs

After the enrichment analysis of the upregulated DEGs, we immediately analyzed the downregulated DEGs. The results in Figure 3(a) displayed that the downregulated DEGs were enriched in BP, such as positive regulation of nitric-oxide synthase biosynthetic process and T cell activation, regulation of nitric-oxide synthase biosynthetic process, and cellular response to fatty acid. In CC, these DEGs were associated with sodium: potassium-exchanging ATPase complex, acrosomal membrane, cytoplasmic side of endoplasmic reticulum membrane, etc. In MF, these DEGs were related to 5′-deoxyribose-5-phosphate lyase activity, androsterone dehydrogenase activity, clathrin heavy chain binding, etc. The KEGG enrichment results in Figure 3(b) demonstrated the first 9 pathways enriched by DEGs were namely malaria, protein digestion and absorption, graft-versus-host disease, cholesterol metabolism, histidine metabolism, cardiac muscle contraction, proximal tubule bicarbonate reclamation, cAMP signaling pathway, and bile secretion.

### 3.4. GSEA

To explore the function of genes in the sample, we used GSEA to analyze the enrichment of genes in BP and set *P* < 0.05 as the selection condition. Figures 4(a)–4(d) show that the genes in 68 samples were significantly enriched in lipid digestion, defense response to fungus, intestinal lipid absorption, and positive regulation of potassium ion transmembrane transporter activity.

### 3.5. Screening of Hub Genes from the PPI Network

According to the Cytoscape software on the STRING website, we constructed a PPI network of DEGs, which contained 215 nodes and 297 edges (Figure 5). The edges between nodes represented the interactions among these genes. In order to screen out the hub genes, we screened out 5 hub genes according to the degrees, namely, CDH1, TFRC, CCL2, BUB1B, and CD19. Among them, CDH1 had the highest degree value of 17, and the other four hub genes had degree values of 12.

### 3.6. Analysis of Hub Gene Expression

In order to further clarify the functions of these 5 hub genes in VAD, we drew a violin chart to compare the levels of hub genes between the control and the VAD groups. According to the results in Figure 6, the expression levels of BUB1B, CCL2, CDH1, and TFRC were higher in the control group. On the contrary, CD19 was highly expressed in the VAD group.

## 4. Discussion

HF is more common in the elderly population, and the prognosis is poor [17]. It causes patients to reduce or lose their ability to take care of themselves and brings a heavy economic burden to patients, family, and society [18]. According to reports, the hospitalization rate of HF patients over 65 years old has risen sharply [19]. As the age of patients aged 65 to 85 increases every 10 years, the incidence of HF in men has doubled, while the incidence in women has tripled. For people 85 years of age or older, the incidence of HF is as high as 13.01 per 1,000 people per year [20]. Based on different standards, HF can be divided into different types. According to the location of HF, it can be divided into left, right, and total HF [21]. According to the ejection fraction, it can be divided into low-volume and high-volume HF or systolic HF and diastolic HF [22]. Here, the gene set GSE21610 analyzed the gene expression patterns of 30 paired samples from VAD supported and 8 nonfailure control hearts.

According to the results of GO and KEGG analysis results, we found G protein-coupled receptor binding, peroxisome, and cAMP signaling pathway were mostly signal pathways of HF. Gaidarov et al. found that the G protein-coupled receptor (GPCR) superfamily of integral membrane proteins was composed of 1,000 members and included 3% of the human genome. Internalization of agonist-activated GPCR is regulated by nonvisual arrestins. It binds to clathrin and is therefore considered an adaptor during endocytosis [23]. The peroxisome proliferator-activated receptor (PPAR) is a ligand-activated transcription factor, which converts the lipid signal into a physiological response by activating the metabolic target gene [24]. Ishiguro et al. proposed that the heart cell cycle 3′,5′-adenosine monophosphate (CAMP) regulates various processes, such as pulsation, contraction, metabolism, and apoptosis [25]. CAMP is the main second messenger of many organs; especially in the heart, it regulates calcium and many other physiological processes: homeostasis, beating frequency, myocardial contractility, and cell death [26]. This mitochondrial CAMP pathway may have clinical significance for HF, because mitochondrial metabolism and CAMP signaling in patients diagnosed with HF are significantly impaired, which is one of the reasons for cardiomyocyte dysfunction [27].

GSEA showed that the gene set was gathered in lipid digestion, defense response to fungus, intestinal lipid absorption, and positive regulation of potassium ion transmembrane transporter activity. Rose et al. proposed that rabbit's APD was prolonged in pacing-induced HF due to a decrease in potassium current densities. Action potential (AP) prolongation is a sign of myocardial failure. The functional downregulation of potassium current is a distinctive feature of ventricular failure cells. The specific changes in potassium expression depend on the type and area of the heart and the process that induces HF [28].

We built a PPI network of DEGs in HF based on the Cytoscape software. Finally, we got five hub genes of HF, and they were CDH1, TFRC, CCL2, BUB1B, and CD19. Previous studies have found that CDH1 encodes a classic cadherin in the cadherin superfamily. The protein is processed to produce mature glycoprotein [29]. CDH1 mutations are associated with gastric cancer, breast cancer, colorectal cancer, thyroid cancer, and ovarian cancer. The loss of function of this gene is believed to promote cancer progression [30]. Huang et al. concluded that TFRC was an important participant in intracellular iron transport [31]. Several reports have shown that certain human tumors, such as anaplastic thyroid cancer and astrocytic brain tumors, have abnormal TFRC overexpression. TFRC enhances the proliferation and metastasis of cancer, thereby promoting the progress of cancer, showing the potential of TFRC as a new therapeutic target for human cancer [32]. The article by Zhang et al. suggested that chemokines were a type of small cytokines that guided a variety of immune/inflammatory cells into the tumor site during tumorigenesis [33]. Abnormal expression of chemokines is related to different types of cancers, including prostate cancer. CCL2 is a chemokine of monocytes/macrophages, B cells, and T lymphocytes and belongs to the CC subfamily of chemokines. CCL2 is highly expressed in plasma, synovial fluid, and synovial tissue previously reported in the literature [34].

## 5. Conclusion

To sum up, the present study has successfully determined the hub genes and pathways in HF progression. Functional and enrichment results show DEGs are significantly enriched in G protein-coupled receptor binding, peroxisome, and cAMP signaling pathway. GSEA suggests that the gene set GSE21610 is concentrated in lipid digestion, defense response to fungus, and intestinal lipid absorption. We also identify that some hub genes (CDH1, TFRC, CCL2, BUB1B, and CD19) are linked with HF. Meanwhile, these hub genes and key pathways are independent prognostic factors for HF. Nevertheless, further studies are needed to confirm the findings in this research.

## Figures and Tables

**Figure 1:** Analysis of volcano diagrams of 8 groups of controls and 30 paired samples of VAD.

**Figure 2:** Functional enrichment analysis of upregulated DEGs. (a) GO analysis. Green represents BP, orange represents CC, and purple represents MF. (b) KEGG pathway. The size of the dot represents the number of enriched genes.

**Figure 3:** Functional enrichment analysis of downregulated DEGs. (a) GO analysis. Green represents BP, orange represents CC, and purple represents MF. (b) KEGG pathway. The size of the dot represents the number of enriched genes.

**Figure 4:** Functional analysis of BP using GSEA. (a) Lipid digestion. (b) Defense response to fungus. (c) Intestinal lipid absorption. (d) Positive regulation of potassium ion transmembrane transporter activity.

**Figure 5:** The PPI network of DEGs and the selection of hub genes. The PPI network of DEGs is established by Cytoscape, and the hub genes are marked with red nodes.

**Figure 6:** Violin chart. Comparison of the expression levels of BUB1B, CCL2, CD19, CDH1, and TFRC in the control group and the VAD group. Blue represents the control group, and pink represents the VAD group. ^∗∗^*P* < 0.01 and ^∗∗∗^*P* < 0.001.

## Data Availability

The datasets used and/or analyzed during the current study are available from the corresponding author on reasonable request.
